The article "Conservative Therapy vs. Endovascular Approach for Intracranial Vertebrobasilar Artery Trunk Large Aneurysms: A Prospective Multicenter Cohort Study" was retracted in 2023. Reasons: signs of a paper mill; suspected computer-generated content; unreliable results or conclusions; lack of ethics approval or compliance.

# Conservative Therapy vs. Endovascular Approach for Intracranial Vertebrobasilar Artery Trunk Large Aneurysms: A Prospective Multicenter Cohort Study

**DOI:** 10.1155/2022/9682507

**Published:** 2022-06-20

**Authors:** Qiaowei Wu, Tianxiao Li, Weijian Jiang, Juha Antero Hernesniemi, Li Li, Yingkun He

**Affiliations:** ^1^Cerebrovascular Department of Interventional Center, Zhengzhou University People's Hospital, Henan University People's Hospital and Henan Provincial People's Hospital, Zhengzhou, Henan, China; ^2^Department of Neurosurgery, The First Affiliated Hospital of Harbin Medical University, Harbin, Heilongjiang, China; ^3^Department of Vascular Neurosurgery, Chinese People's Liberation Army Rocket Force Characteristic Medical Center, Beijing, China

## Abstract

**Background:**

Intracranial vertebrobasilar trunk large (≥10 mm) aneurysms (IVBTLAs) are rare and challenging to manage. In this study, we describe the natural prognosis and evaluate the safety and efficacy of endovascular treatment of IVBTLAs compared with conservative therapy.

**Methods:**

This prospective multicenter cohort study included patients with IVBTLAs, who chose either endovascular treatment (endovascular group) or conservative therapy (conservative group) after discussion with their doctors. The primary endpoint was the incidence of serious adverse events (SAEs) related to the target vessel, while secondary endpoints included target vessel-related mortality, major stroke, other serious adverse events, and aneurysm occlusion rate.

**Results:**

In total, 258 patients were referred to our two centers for the management of vertebrobasilar aneurysms, and 69 patients had IVBTLAs. Among them, 51 patients underwent endovascular treatment, and 18 patients received conservative therapy. The incidence of target vessel-related SAEs was 15.7% (8/51) in the endovascular group and 44.4% (8/18) in the conservative group (*P* = 0.031). The target vessel-related mortality was 2.0% (1/51) in the endovascular group and 38.9% (7/18) in the conservative group (*P* < 0.001). The cumulative survival rates in the endovascular group and conservative group within 1-year, 3-year, and 5-year were 98.0% vs. 83.3%, *P* = 0.020; 98.0% vs. 66.7%, *P* = 0.001; and 98.0% vs. 35.6%, *P* < 0.001, respectively. Multivariate analysis revealed conservative therapy, giant aneurysm, and ischemic onset as risks factor for SAEs.

**Conclusions:**

Compared with conservative treatment, endovascular treatment of the IVBTLAs may be associated with a lower incidence of SAEs, with higher 1-year, 3-year, and 5-year survival rates. Conservative therapy, giant aneurysm, and ischemic onset were associated with a high risk of SAEs.

The article "Conservative Therapy vs. Endovascular Approach for Intracranial Vertebrobasilar Artery Trunk Large Aneurysms: A Prospective Multicenter Cohort Study" was retracted in 2023. Reasons: signs of a paper mill; suspected computer-generated content; unreliable results or conclusions; lack of ethics approval or compliance.

## 1. Introduction

The intracranial vertebrobasilar trunk artery is defined as the arterial segment extending from the origin of the intracranial vertebral artery up to the origin of the superior cerebellar artery. Aneurysms originating from the branch of the vertebrobasilar artery and basilar tip aneurysms are excluded from intracranial vertebrobasilar trunk aneurysms [1]. Endovascular treatment is the most commonly used method for treatment of these aneurysms, which have always posed a great challenge to physicians due to their location, pathological features, relation to perforating branches of the vertebrobasilar artery, higher risks of procedural complications, and poorer outcomes compared with anterior circulation aneurysms [2–5]. According to published studies, aneurysms could be defined as small aneurysms (<10 mm in maximum diameter), large aneurysms (10 to <25 mm), and giant aneurysms (≥25 mm) [6, 7]. As intracranial vertebrobasilar trunk large (≥10 mm) aneurysms (IVBTLAs) rarely occur, there are limited data on the epidemiology, natural history, and management, besides case reports [1, 8–10]. The natural prognosis of IVBTLAs and the safety and efficacy of endovascular treatment still need to be further confirmed. Therefore, this study was conducted to explore the natural prognosis of conservative therapy and the safety and efficacy of endovascular treatment of IVBTLAs.

## 2. Materials and Methods

### 2.1. Study Design and Participants

This prospective multicenter cohort study of conservative therapy versus endovascular approach for IVBTLAs was conducted in Henan Provincial People's Hospital and Chinese People's Liberation Army Rocket Force Characteristic Medical Center between October 2012 and October 2018. The date of follow-up was ended in March 2019. The institutional review board of the lead center (Henan Provincial People's Hospital) approved the study (No. 12072), and the ethics approval documents were recorded and registered in Chinese People's Liberation Army Rocket Force Characteristic Medical Center. The study was carried out in accordance with the 1964 Declaration of Helsinki. Informed consent was obtained from the patients before the enrollment of the study, and the treatment decision was made. The doctors informed the patients of all treatment options, after which the patients individually discussed with their doctors and chose endovascular treatment (endovascular group) or refused to receive further surgical treatment (conservative group).

The major criterion for inclusion in the study was aneurysm arising from the intracranial vertebrobasilar trunk artery, measuring ≥10 mm in diameter and modified Rankin Scale (mRS) ≤ 2 before the symptom onset. The major cause for exclusion was an aneurysm involving the extracranial segment of vertebral artery, basilar tip, and superior cerebellar artery aneurysms, complicated by other intracranial aneurysms. Patients with vertebrobasilar dolichoectasia were also excluded. Patients' inclusion and exclusion criteria are detailed in Supplemental Table 1.

The article "Conservative Therapy vs. Endovascular Approach for Intracranial Vertebrobasilar Artery Trunk Large Aneurysms: A Prospective Multicenter Cohort Study" was retracted in 2023. Reasons: signs of a paper mill; suspected computer-generated content; unreliable results or conclusions; lack of ethics approval or compliance.

### 2.2. Endovascular Treatment

The endovascular strategies for all patients in the endovascular group can be divided into 3 following techniques: reconstructive technique, deconstructive technique, and combination therapy.

#### 2.2.1. Reconstructive Technique

The reconstructive technique included coiling, stent-assisted coiling, and flow diversion (FD). The parent artery maintained patency after the procedure. The technique was mostly used in patients with saccular aneurysms, patients with insufficient collateral circulation, or other aneurysms at the discretion of the neurointerventionists. The procedures were performed under general anesthesia and systemic heparinization (50–70 U/kg). After sheath placement, a suitable guiding catheter was placed in the distal vertebral artery. Three-dimensional (3D) rotational angiography was performed, and 3D reconstruction was used to determine the work projection, measure the parent artery and aneurysms, and determine the treatment protocol. Depending on operator preferences, aneurysms were coiled with stent-assisted by LVIS (MicroVention-Terumo, California, USA), Enterprise (Codman Neurovascular, Massachusetts, USA), Solitaire (ev3, Irvine, California, USA), and LEO (Balt, Montmorency, France). A Pipeline embolization device (Covidien, Irvine, California, USA) was used for patients with FD treatment.

#### 2.2.2. Deconstructive Technique

The deconstructive technique included parent artery sacrifice and aneurysm embolization combined with parent artery sacrifice. Preliminary digital subtraction angiography (DSA) with a collateral circulation test and a balloon occlusion test (BOT) under local infiltration anesthesia and systemic heparinization was performed before the procedure. The balloon was placed in the proximal parent artery. In addition, prior to balloon inflation, the mean arterial pressure was pharmacologically decreased by a third, in order to maximize the sensitivity of the BOT. After the balloon inflation, a 30 min observation was maintained [11]. If the neurological status remained unchanged during the BOT, the aneurysm occlusion and parent artery sacrifice were performed using coils.

#### 2.2.3. Reconstruction and Deconstruction Combined Technique

The combined technique of reconstruction and deconstruction incorporated the characteristics of the two methods, where reconstruction therapy ensured the unobstructed parent artery, and unilateral vertebral artery sacrificing reduced the blood flow to the aneurysm.

The article "Conservative Therapy vs. Endovascular Approach for Intracranial Vertebrobasilar Artery Trunk Large Aneurysms: A Prospective Multicenter Cohort Study" was retracted in 2023. Reasons: signs of a paper mill; suspected computer-generated content; unreliable results or conclusions; lack of ethics approval or compliance.

### 2.3. Antiplatelet Therapy

For patients with unruptured aneurysms who underwent reconstructive therapy or combined therapy, daily dual antiplatelet therapy (75 mg clopidogrel and 100 mg aspirin) was prescribed for at least 3-5 days before the procedural. For patients with ruptured aneurysms, a loading dose of 300 mg clopidogrel and 300 mg aspirin or tirofiban (intravenous bolus (8 *μ*g/kg) over 3 min followed by a maintenance dose of 0.1 mg/kg/min for 24-48 h) was administrated [12, 13]. At least 3 days after the dual antiplatelet administration, thromboelastography (TEG) was used to evaluate the platelet function. For clopidogrel hyporesponders, the clopidogrel would be changed to ticagrelor 90 mg, twice daily. Daily antiplatelet therapy (75 mg clopidogrel and 100 mg aspirin) was maintained for at least 3 months, while 100 mg aspirin was continued indefinitely.

### 2.4. Conservative Therapy

Conservative therapy was divided into 2 strategies: antiplatelet therapy and risk factors control. For patients with ischemic onset, the daily antiplatelet agent was used (75 mg clopidogrel or 100 mg aspirin) infinitely. TEG was also used to test the platelet function, and for clopidogrel hyporesponders, the clopidogrel would be changed to ticagrelor. In addition, risk factors such as hypertension, diabetes, and smoking were controlled. Patients with hemorrhage or other onset were treated by controlling risk factors. Daily blood pressure and blood glucose measurements were instructed to all the patients with hypertension and diabetes to ensure the modification.

### 2.5. Follow-Up

Patients underwent clinical assessments at day 1, day 7, day 30, 6 months, 1 year, and annual follow-up postprocedure. Imaging follow-up (DSA or MR) was performed at 6 months postprocedure. All clinical and imaging data were submitted for assessment by an independent laboratory. Investigators were requested to report all adverse events and to judge the relationship to the target vessel. Ischemic stroke was evaluated by the National Institute of Health Stroke Scale (NIHSS); NIHSS increase < 6 was defined as minor stroke, while NIHSS increase ≥ 6 was defined as major stroke. Clinical outcomes were evaluated by mRS, and mRS ≤ 2 was defined as a good outcome. The degree of aneurysm occlusion status was evaluated according to the Roy–Raymond grading scale [14].

### 2.6. Study Endpoints

The primary endpoint was the incidence of serious adverse events (SAEs) related to the target vessel, which included death, thromboembolic events (partial or complete occlusion of parent artery on DSA or thromboembolism symptoms with or without cerebral infarction on postprocedural MRI/CT), hemorrhagic events (new intracranial hemorrhage on postprocedural head CT/MRI with or without certain clinical symptoms), or other threatening events, leading to hospitalizations or prolonged hospitalizations. Secondary endpoints included target vessel-related mortality, major stroke (ischemic or hemorrhagic), other SAEs, and aneurysm occlusion rate.

The article "Conservative Therapy vs. Endovascular Approach for Intracranial Vertebrobasilar Artery Trunk Large Aneurysms: A Prospective Multicenter Cohort Study" was retracted in 2023. Reasons: signs of a paper mill; suspected computer-generated content; unreliable results or conclusions; lack of ethics approval or compliance.

### 2.7. Statistical Analysis

Statistical analysis was performed using SPSS 22.0 software (IBM SPSS Inc., Chicago, IL, USA) by independent statisticians. Continuous variables were presented as mean ± SD, median, and interquartile range (IQR). Qualitative variables were presented as numbers followed by percentages. Independent-sample *t*-test, chi-square test, and Fisher's exact test were used to verify the differences between variables. Kaplan-Meier survival analysis was used to compare the cumulative incidence of SAEs and death in the endovascular and conservative groups. Univariate and multivariate Cox regression analysis was performed to identify the independent risk factors for SAEs. *P* < 0.05 was considered as statistically significant.

## 3. Results

### 3.1. Patients' Characteristics

Between October 2012 and October 2018, a total of 258 patients were referred to our two centers for the management of vertebrobasilar aneurysms, and 69 patients were enrolled in our study (Figure 1). The cohort comprised 48 (69.6%) males and 21 (30.4%) females, with a median age of 56.0 years (IQR, 47.5-62.5). The maximal median diameter of the aneurysms was 14.8 mm (IQR, 12.0-20.0). Most aneurysms were located in the basilar artery (*n* = 27, 39.1%), followed by vertebral artery (*n* = 26, 37.7%), and vertebrobasilar junction (*n* = 16, 23.2%). Among the 69 patients, 51 underwent the endovascular treatment (endovascular group), and 18 received the antiplatelet and (or) risk factors control treatment (conservative group). The conservative group had higher rates of hypertension and giant aneurysms compared to the endovascular group (94.4% vs. 64.7%, *P* = 0.034; 50.0% vs. 19.6%, *P* = 0.030). Detailed baseline patient and aneurysm characteristics are shown in Table 1.

Of the 51 patients in the endovascular group, 36 (70.6%) underwent the reconstructive treatment, 11 (21.6%) underwent the deconstructive treatment, and 4 (7.8%) underwent the combined treatment. Detailed procedure-related data are shown in Table 2. In the conservative group, 11 (61.1%) patients received the risk factor control, and 7 (38.9%) received the antiplatelet and risk factor control treatment.

The article "Conservative Therapy vs. Endovascular Approach for Intracranial Vertebrobasilar Artery Trunk Large Aneurysms: A Prospective Multicenter Cohort Study" was retracted in 2023. Reasons: signs of a paper mill; suspected computer-generated content; unreliable results or conclusions; lack of ethics approval or compliance.

### 3.2. Primary Endpoint

The clinical follow-up was available for all the 69 patients, with a median of 34.0 (IQR, 6.5-47.5) months. The incidence of all SAEs associated with the target vessel was 15.7% (8/51) in the endovascular group and 44.4% (8/18) in the conservative group (RR = 0.35, 95% CI, 0.16-0.80; *P* = 0.031). The proportion of cases with good outcomes (mRS ≤ 2) in the endovascular group was higher than that in the conservative group (88.2% vs. 55.6%, *P* = 0.009) (Table 3).

Among 8 patients with SAEs in the endovascular group, 4 had ischemic symptoms with the final mRS of 3, 3, 4, and 4, respectively. Transient ischemic symptoms were found in 3 patients with the final mRS of 1, 0, and 0, respectively. One patient suffered subarachnoid hemorrhage (SAH) 3 months after the procedure and subsequently died (Supplemental Figure 1). Among 8 patients with SAEs in the conservative group, 4 died due to the aneurysm rupture. One patient died due to brainstem compression, and 2 due to an ischemic stroke. The remaining patient had persistent ischemic symptoms and a final mRS of 1.

### 3.3. Other Outcomes

During the follow-up, significantly lower mortality was found in the endovascular group compared to the conservative group (2.0% vs. 38.9%, *P* < 0.001). The proportion of patients with hemorrhagic stroke was also higher in the conservative group (2.0% vs. 22.2%, *P* = 0.020). The proportion of patients with ischemic stroke was similar between the endovascular group and conservative group (13.7% vs. 16.7%, *P* = 1.000). Fifty-three imaging follow-ups were analyzed at a median of 6.0 (IQR, 6.0-12.5) months, revealing 56.8% (25/44) of the aneurysms in the endovascular group with complete occlusion (Supplemental Figure 2), while no aneurysms occluded (0/9) in the conservation group. The detailed outcomes are described in Table 3.

### 3.4. Survival Analysis

The 1- and 3-year SAE-free cumulative survival rates of patients in the endovascular group were similar to those in the conservative group (88.2%, 95% CI: 29.5% to 99.3% vs. 76.9%, 95% CI: 18.8% to 97.9%, *P* = 0.322; 85.5%, 95% CI: 28.7% to 98.9% vs. 61.5%, 95% CI: 13.1% to 94.4%, *P* = 0.085). The 5-year SAE-free cumulative survival rate of patients in the endovascular group was higher compared to that in the conservative group (85.5%, 95% CI: 28.7% to 98.9% vs. 32.8%, 95% CI: 3.1% to 88.1%, *P* = 0.007) (Figure 2). Also, the 1-year, 3-year, and 5-year overall cumulative survival rates of patients in the endovascular group were higher than those in the conservative group (98.0%, 95% CI: 19.5% to 99.9% vs. 83.3%, 95% CI: 20.4% to 99.0%, *P* = 0.020; 98.0%, 95% CI: 19.5% to 99.9% vs. 66.7%, 95% CI: 14.5% to 95.9%, *P* = 0.001; and 98.0%, 95% CI: 19.5% to 99.9% vs 35.6%, 95% CI: 3.6% to 89.2%, *P* < 0.001) (Figure 2, Supplemental Table 2).

The article "Conservative Therapy vs. Endovascular Approach for Intracranial Vertebrobasilar Artery Trunk Large Aneurysms: A Prospective Multicenter Cohort Study" was retracted in 2023. Reasons: signs of a paper mill; suspected computer-generated content; unreliable results or conclusions; lack of ethics approval or compliance.

### 3.5. Subgroup Analysis

There was no significant difference (*P* = 1.000) in the overall SAEs between constructive treatment (5/36, 13.9%) and deconstructive treatment (1/11, 9.1%). For patients with unruptured aneurysms, the incidence of overall SAEs in the endovascular group was lower than that in the conservative group (7/43, 16.3% vs 8/18, 44.4%, *P* = 0.045). For patients treated with reconstructive techniques, stent-assisted coiling showed a higher complete aneurysm occlusion rate compared with sole stenting or sole FD implantation (13/24, 54.2% vs 0/7, 0%, *P* = 0.025). Deconstructive treatment was associated with high rates of complete occlusion of aneurysms in comparison to reconstructive treatment (10/10, 100% vs. 13/31, 41.9%, *P* = 0.004).

### 3.6. Risk Factors of SAEs

Univariate analysis showed that ischemic onset (*P* = 0.006), aneurysms involving basilar artery (*P* = 0.054), giant aneurysms (*P* = 0.011), and conservative treatment (*P* = 0.002) were related to SAEs. Multivariate analysis revealed fewer SAEs in the endovascular group than in the conservative group (HR = 4.42, 95% CI: 1.48 to 13.19; *P* = 0.008). Also, ischemic onset (HR = 3.33, 95% CI: 1.19 to 9.32; *P* = 0.022) and giant aneurysms (HR = 2.85, 95% CI: 1.01 to 8.04; *P* = 0.049) resulted as statistically significant risk factors associated with SAEs after controlling for fusiform and/or dissecting aneurysms and aneurysms involved basilar artery (Table 4).

## 4. Discussion

Currently, there are limited reports on the epidemiology of IVBTLAs. Previous studies have shown that the percentage of vertebrobasilar or posterior cerebral artery aneurysms (basilar tip aneurysms were not included) among the overall aneurysm locations is 6.6% [6], with an overall dismal prognosis after the aneurysm rupture [5]. In addition, Mizutani et al. [15] reported that the recurrent rupture rate of untreated ruptured vertebrobasilar was 71.4%, and it most commonly occurred within 24 hours after the first rupture, resulting in a mortality of 46.7%. Due to the high risk of rupture and poor natural history of IVBTLAs, once detected, it is important to individualize surgical intervention on the basis of the patient's overall medical condition, and aneurysm obliteration should be performed as soon as the patient is medically stabilized because of rebleeding [15]. In our study, the mortality of the conservative group was 38.9% (7/18), where 4 (4/7, 57.1%) cases were due to ruptured aneurysms.

The anatomy location and pathological feature of large vertebrobasilar aneurysms, such as the limited surgical accessibility and the relation to perforating branches, limit open surgical options, including clipping, wrapping, vessel occlusion, and bypass, which are often associated with high morbidity and mortality [16, 17]. Endovascular treatment has been increasingly used for treating such aneurysms, which can avoid the extensive surgical invasion and cranial nerve deficits associated with open surgery [2, 16, 18]. In this study, the overall target vessel-related SAE rate in the endovascular group was 15.7%, which was significantly lower compared to that in the conservative group. Especially low mortality (2.0%) and hemorrhagic stroke rate (2.0%) were also observed. Endovascular therapy can be divided into two methods according to different therapeutic concepts: (1) aneurysm treated by coiling, stent-assisted coiling, or FD (reconstructive treatment) and (2) parent artery sacrifice (deconstructive treatment). In specific cases, it is also possible to combine these two methods. BOT is necessary before the deconstructive treatment so as to avoid severe ischemic stroke after occlusion, especially fatal brainstem ischemia. Parent artery sacrifice should only be considered if the collateral circulation is good. Nevertheless, patients with a negative BOT are still at risk for ischemia, and sometimes, bypass procedures are needed [2, 19, 20]. Then again, a large meta-analysis reported that aneurysms were more likely to be completely occluded after the deconstructive treatment, with the complete occlusion rate which was 93% and 71% after deconstructive and reconstructive treatments, respectively [2]. Another meta-analysis also demonstrated that the deconstructive treatment was associated with higher rates of complete aneurysmal occlusion compared with reconstructive treatment (88.0% vs. 81.0%) [21]. In the present study, the complete occlusion rate was 100% without an increase in ischemic complications.

The article "Conservative Therapy vs. Endovascular Approach for Intracranial Vertebrobasilar Artery Trunk Large Aneurysms: A Prospective Multicenter Cohort Study" was retracted in 2023. Reasons: signs of a paper mill; suspected computer-generated content; unreliable results or conclusions; lack of ethics approval or compliance.

With the development of new intracranial stents, reconstructive treatments of large intracranial aneurysms have become more widely used, especially in patients with insufficient collateral circulation [2, 22, 23]. However, single stenting or series stenting of IVBTLAs cannot completely obliterate the aneurysm sac. In our study, 2 cases underwent the single stenting, and 4 underwent the series stenting; however, all the aneurysms remained unchanged during the follow-up. The concomitant coiling was needed to facilitate the aneurysmal occlusion and prevent the rupture of aneurysms. For large or giant vertebrobasilar aneurysms treated with stent-assisted coiling, Li et al. [24] reported a recurrence rate of 33.3%, while Mu and colleagues [25] reported a recanalization rate of 66.6%, with a complication rate of 36.4%. In our study, the complete occlusion rate was 54.2% during the follow-up after stent-assisted coiling, and the SAE rate was 15.4%, including mortality of 3.9%. Over recent years, FD has been used as a reconstructive option. In the present study, only a few patients were treated with FD, and the long-term results remain to be observed. Nonetheless, previous studies have shown promising results after FD treatment of intracranial vertebrobasilar aneurysms [22, 26–28]. Kumar et al. [27] compared the long-term imaging outcomes of intradural vertebral artery aneurysms following parent artery sacrifice or FD treatment, revealing a complete occlusion rate of 81.5% in the FD group and comparable intraprocedural complications and long-term clinical and imaging outcomes. Bhogal et al. [28] reported a case series of 56 nonsaccular posterior circulation aneurysms (mean diameter = 11 mm) treated with FD, with a complete occlusion rate of 75% in fusiform aneurysms and an overall complication rate of 15.5%.

In the present study, we found a significantly lower SAE rate in the endovascular group compared to the conservative group (15.7% vs. 44.4%, *P* = 0.031). In the endovascular group, 7 (13.7%) patients presented with procedure-related ischemic stroke, and there was 1 (2.0%) death case. The specific reasons for the 7 ischemic strokes are not yet clarified. Of these, 5 out of 7 patients experienced complications within 30 days following the procedure, which may be due to the procedure-related branch vessels or perforator occlusion [29]. In addition, the detachment of parent artery mural thrombus or intraluminal thrombus during the stenting or coiling may also be the potential cause. The other 2 out of 7 patients experienced complications during the follow-up period. Meanwhile, the follow-up DSA revealed that the former dissecting aneurysms were enlarged, and the dissecting lesions that involved vital perforators may be the possible cause. Our study results suggested that giant aneurysms were associated with a high risk of SAEs after managing IVBTLAs. Giant aneurysms often present with intraluminal thrombosis, brainstem compression, and branch vessels or perforator involvement [30, 31]. Patients with giant aneurysms have a higher rate of poor outcomes after surgical or endovascular procedures [5, 30], and giant aneurysms have often been related to a worse natural history, frequently leading to aneurysm rupture, ischemic stroke, and mass effect [5, 6]. Moreover, we found that the ischemic onset was also associated with a high risk of SAEs. Flemming et al. [32] found that the history of prior ischemia was a predictor of cerebral ischemia related to the nonsaccular vertebrobasilar aneurysms. For patients initially presenting with ischemic onset, recurrent ischemic stroke risk was 6.7% per year, with the median time to second ischemic stroke of 1.73 years. The risk of aneurysm-related ischemic stroke was reported to increase from 2.7% at 1 year to 15.9% at 10 years. IVBTLAs are often accompanied by intraluminal thrombus, and the intraluminal thrombus detachment may cause occlusion of perforating vessels or distal vessels, leading to ischemic stroke [33]. The in situ thrombus formation within the parent artery or within perforating vessels may also cause ischemia before and after the aneurysm management.

The article "Conservative Therapy vs. Endovascular Approach for Intracranial Vertebrobasilar Artery Trunk Large Aneurysms: A Prospective Multicenter Cohort Study" was retracted in 2023. Reasons: signs of a paper mill; suspected computer-generated content; unreliable results or conclusions; lack of ethics approval or compliance.

To the best of our knowledge, this is the first study that evaluated the safety and efficacy of endovascular treatment of IVBTLAs compared with conservative therapy in order to gain a better understanding of which management methods might be the most beneficial to the patients. Deconstructive treatment seems to be associated with a higher rate of complete aneurysm occlusion; however, we did not find a significant difference in safety between constructive treatment, deconstructive treatment, and the combined treatment. Therefore, when deconstructive treatment is not feasible, the parent artery reconstruction with various manners can be used as a safe and effective choice.

The present study has some limitations. First, the conservative group had a small sample size, which was insufficient to conclude the natural prognosis of IVBTLAs. In addition, even though the study had a prospective design, due to the selection bias or the insufficient sample size, the baseline characteristics of the two groups were not completely balanced, and there were more giant aneurysms and hypertension patients in the conservative group. Moreover, 16 (23.2%) patients were lost to imaging follow-up, which might impact the evaluation of changes in aneurysms.

## 5. Conclusions

Endovascular treatment of IVBTLAs may be associated with lower rates of SAEs, death, and intracranial hemorrhage as compared with conservative treatment, with high 1-year, 3-year, and 5-year overall cumulative survival rates. Deconstructive treatments led to higher rates of complete occlusion of aneurysms, while stent-assisted coiling showed favorable complete occlusion rates in reconstructive treatments. In addition to conservative treatment, giant aneurysms and ischemic onset could increase the risk of SAEs.

## Figures and Tables

**Figure 1:** Flow chart of the patient selection process.

**Figure 2:** Kaplan–Meier survival curves for SAE-free cumulative survival rates (a) and overall cumulative survival rates (b) according to treatment.

The article "Conservative Therapy vs. Endovascular Approach for Intracranial Vertebrobasilar Artery Trunk Large Aneurysms: A Prospective Multicenter Cohort Study" was retracted in 2023. Reasons: signs of a paper mill; suspected computer-generated content; unreliable results or conclusions; lack of ethics approval or compliance.

**Table 1:** Baseline characteristics of patients and aneurysms.

Characteristics	Endovascular group (*n* = 51)	Conservative group (*n* = 18)	*P* value
Male, *n* (%)	38 (74.5)	10 (55.6)	0.133
Age (years) (IQR)	56.0 (43.0, 62.0)	58.5 (51.0, 66.3)	0.107
Risk factors, *n* (%)			
Hypertension	33 (64.7)	17 (94.4)	0.034
Diabetes mellitus	1 (2.0)	0	1.000
Smoking	11 (21.6)	2 (11.1)	0.532
Family history	1 (2.0)	0	0.739
Onset symptoms, *n* (%)			0.119
Ischemic stroke	12 (23.5)	7 (38.9)	
Hemorrhage	8 (15.7)	0	
Others	31 (60.8)	11 (61.1)	
Aneurysm location, *n* (%)			<0.001
BA	21 (41.2)	6 (33.3)	
VBJ	5 (9.8)	11 (61.1)	
VA	25 (49.0)	1 (5.6)	
Aneurysm shape, *n* (%)			1.000
Saccular	14 (27.5)	5 (27.8)	
Fusiform and/or dissecting	37 (72.5)	13 (72.2)	
Aneurysm's size, *n* (%)			0.030
Large	41 (80.4)	9 (50.0)	
Giant	10 (19.6)	9 (50.0)	
Wide-necked aneurysms, *n* (%)	47 (92.2)	17 (94.4)	1.000
Aneurysms involving side branches, *n* (%)	17 (33.3)	9 (50.0)	0.210

IQR: interquartile range; BA: basilar artery; VBJ: vertebrobasilar junction; VA: vertebral artery.

**Table 2:** Endovascular procedure-related data.

Procedure details	*n* = 51 patients
Catheter access, *n* (%)	51 (100)
Femoral access	47 (92.2)
Radial access	3 (5.9)
Brachial access	1 (2.0)
Reconstructive treatment, *n* (%)	36 (70.6)
Sole stenting	6/36 (16.7)
Single stent	2/6 (33.3)
Series stents	4/6 (66.7)
Stent-assisted coiling	26/36 (72.2)
Single stent-assisted	11/26 (42.3)
Series stent-assisted	15/26 (57.7)
Flow diverter treatment	4/36 (11.1)
Flow diverter alone	2/4 (50)
Adjunct coiling	2/4 (50)
Deconstructive treatment, *n* (%)	11 (21.6)
Reconstruction and deconstruction combined treatment, *n* (%)	4 (7.8)
Stent-assisted coiling and unilateral vertebral artery sacrifice	3/4 (75)
FD implantation and unilateral vertebral artery sacrifice	1/4 (25)
Antiplatelet treatment application after the procedure, *n* (%)	40 (78.4)
Type of stent placed, *n* (%)	*n* = 67 stents
LVIS	22 (32.8)
Enterprise	34 (50.7)
LEO	4 (6.0)
Solitaire	2 (3.0)
Pipeline embolization device	5 (7.5)

**Table 3:** Treatment and imaging outcomes of patients.

Characteristics	Endovascular group	Conservative group	RR (95% CI)	*P* value
Number of patients with clinical FU	51	18	—	—
Median clinical FU (m) (IQR)	39.0 (9.0, 48.0)	19.5 (4.8, 38.3)	—	0.030
Overall SAEs, *n* (%)	8 (15.7)	8 (44.4)	0.35 (0.16-0.80)	0.031
Death	1 (2.0)	7 (38.9)	0.05 (0.01-0.38)	<0.001
Ischemic stroke	7 (13.7)	3 (16.7)	0.82 (0.24-2.8)	1.000
Major stroke	4 (7.8)	2 (11.1)		
Minor stroke	3 (5.9)	1 (5.6)		
Hemorrhage	1 (2.0)	4 (22.2)	0.09 (0.01-0.74)	0.020
Others	2 (3.9)	1 (5.6)	0.71 (0.07-7.33)	1.000
SAEs within 30 d of enrollment^∗^, *n* (%)	6 (11.8)	2 (11.1)	1.06 (0.24-4.78)	1.000
Death	0	2 (11.6)	0.07 (0.01-1.45)	0.065
Ischemic stroke	5 (9.8)	1 (5.6)	1.77 (0.22-14.11)	0.949
Major stroke	2 (3.9)	1 (5.6)		
Minor stroke	3 (5.9)	0		
Hemorrhage	1 (2.0)	1 (5.6)	0.35 (0.02-5.53)	0.457
SAEs 30 d after enrollment^∗^, *n* (%)	4 (7.8)	6 (33.3)	0.24 (0.08-0.74)	0.024
Death	1 (2.0)	5 (27.8)	0.07 (0.01-0.56)	0.004
Ischemic stroke	2 (3.9)	2 (11.6)	0.35 (0.05-2.32)	0.592
Major stroke	2 (3.9)	1 (5.6)		
Minor stroke	0	1(5.6)		
Intracranial hemorrhage	1 (2.0)	3 (16.7)	0.12 (0.01-1.06)	0.086
Others	1 (2.0)	1 (5.6)	0.35 (0.02-5.35)	0.457
mRS at last follow-up, *n* (%)			—	0.009
0-2	45 (88.2)	10 (55.6)		
3-6	6 (11.8)	8 (44.4)		
Number of patients with imaging FU	44	9		
Median imaging FU (m) (IQR)	6.0 (6.0, 12.0)	12.0 (12.0, 22.0)		
Aneurysm imaging finding, *n* (%)			—	<0.001
Occluded	25 (56.8)	0		
Improved	3 (6.8)	0		
Stable	9 (20.5)	5 (55.6)		
Recanalized	5 (11.4)	0		
Enlarged	2 (4.5)	4 (44.4)		

FU: follow-up; IQR: interquartile range; SAEs: serious adverse events; mRS: modified Rankin Scale. ^∗^One patient experienced two intracranial hemorrhage events, one within 30 days of enrollment and one 30 days after enrollment. One patient experienced a minor stroke within 30 days and an SAE (gross hematuria) after 30 days. One patient had a major stroke within 30 days and a minor stroke after 30 days.

The article "Conservative Therapy vs. Endovascular Approach for Intracranial Vertebrobasilar Artery Trunk Large Aneurysms: A Prospective Multicenter Cohort Study" was retracted in 2023. Reasons: signs of a paper mill; suspected computer-generated content; unreliable results or conclusions; lack of ethics approval or compliance.

**Table 4:** Univariable and multivariable analysis for serious adverse events.

Variable	Univariable			Multivariable		
	HR	95% CI	*P* value	HR	95% CI	*P* value
Conservative treatment	5.40	1.84-15.90	0.002	4.42	1.48-13.19	0.008
Aneurysms involving side branches	0.90	0.33-2.47	0.844	—	—	—
Aneurysm's size (≥25 mm)	3.72	1.35-10.22	0.011	2.85	1.01-8.04	0.049
Fusiform and/or dissecting aneurysms	0.52	0.15-1.85	0.316	1.90	0.50-7.29	0.348
Age (>60 years)	1.63	0.59-4.52	0.344	—	—	—
Sex (male)	1.00	0.34-2.94	0.998	—	—	—
Aneurysms involved basilar artery	3.51	0.98-12.62	0.054	2.42	0.49-11.96	0.280
Hypertension	2.34	0.52-10.46	0.226	—	—	—
Ischemic onset	4.21	1.51-11.71	0.006	3.33	1.19-9.32	0.022
Ruptured aneurysms	0.411	0.05-3.16	0.411	—	—	—
Diabetes mellitus	0.76	0.17-3.39	0.720	—	—	—
Smoking	0.37	0.05-2.85	0.341	—	—	—

## Data Availability

Unpublished data are available upon reasonable request from the corresponding author.

## Supplementary Materials

Supplementary Materials Supplemental Table 1: summary of inclusion and exclusion criteria. Supplemental Table 2: survival analysis results. Figure 1: (A) pretreatment anteroposterior DSA showing a basilar giant saccular aneurysm. (B) High-resolution magnetic resonance-enhanced scanning showing the aneurysm wall was enhanced (arrow). (C) Double LVIS stent-assisted coiling was performed; the immediate postprocedural DSA showing the aneurysm sac was completely occluded. (D) The patient presented with severe headaches the second day after the procedure, and the emergency head CT showed the subarachnoid hemorrhage. (E) The followed DSA showing that the coils were compressed. (F) Additional double enterprise stent-assisted coiling was performed. The patient died of aneurysm rerupture 2 months after discharge. Figure 2: (A, B) pretreatment anteroposterior DSA (A) three-dimensional construction (B) showing a vertebrobasilar junction giant saccular aneurysm. (C) Magnetic resonance image revealed severe brain stem compression. (D) Enterprise stent-assisted coiling was performed; the immediate postprocedural DSA showing the embolization result (E). (F) The follow-up DSA at 6 months demonstrated that the aneurysm was completely occluded.

The article "Conservative Therapy vs. Endovascular Approach for Intracranial Vertebrobasilar Artery Trunk Large Aneurysms: A Prospective Multicenter Cohort Study" was retracted in 2023. Reasons: signs of a paper mill; suspected computer-generated content; unreliable results or conclusions; lack of ethics approval or compliance.

## References

[1] Saliou G., Sacho R. H., Power S. (2015). Natural history and management of basilar trunk artery aneurysms. *Stroke*.

[2] Cagnazzo F., Mantilla D., Rouchaud A. (2018). Endovascular treatment of very large and giant intracranial aneurysms: comparison between reconstructive and deconstructive techniques-a meta-analysis. *American Journal of Neuroradiology*.

[3] Fang Y. B., Lin A., Kostynskyy A. (2018). Endovascular treatment of intracranial vertebrobasilar artery dissecting aneurysms: parent artery occlusion versus flow diverter. *European Journal of Radiology*.

[4] Wang J., Jia L., Yang X. (2019). Outcomes in symptomatic patients with vertebrobasilar dolichoectasia following endovascular treatment. *Frontiers in Neurology*.

[5] Wiebers D. O., Whisnant J. P., Huston J 3rd (2003). Unruptured intracranial aneurysms: natural history, clinical outcome, and risks of surgical and endovascular treatment. *The Lancet*.

[6] Investigators ISoUIA (1998). Unruptured intracranial aneurysms — risk of rupture and risks of surgical intervention. *The New England Journal of Medicine*.

[7] Wiebers D. O. (2006). Unruptured intracranial aneurysms: natural history and clinical management. Update on the international study of unruptured intracranial aneurysms. *Neuroimaging Clinics of North America*.

[8] Chung J., Park H., Lim Y. C., Hyun D. K., Shin Y. S. (2011). Endovascular treatment of basilar artery trunk aneurysms. *Acta Neurochirurgica*.

[9] Higa T., Ujiie H., Kato K., Kamiyama H., Hori T. (2009). Basilar artery trunk saccular aneurysms: morphological characteristics and management. *Neurosurgical Review*.

[10] Zhang Y., Zhou Y., Yang P. (2016). Comparison of the flow diverter and stent-assisted coiling in large and giant aneurysms: safety and efficacy based on a propensity score-matched analysis. *European Radiology*.

The article "Conservative Therapy vs. Endovascular Approach for Intracranial Vertebrobasilar Artery Trunk Large Aneurysms: A Prospective Multicenter Cohort Study" was retracted in 2023. Reasons: signs of a paper mill; suspected computer-generated content; unreliable results or conclusions; lack of ethics approval or compliance.

[11] Lesley W. S., Rangaswamy R. (2009). Balloon test occlusion and endosurgical parent artery sacrifice for the evaluation and management of complex intracranial aneurysmal disease. *Journal of NeuroInterventional Surgery*.

[12] Liang X. D., Wang Z. L., Li T. X. (2016). Safety and efficacy of a new prophylactic tirofiban protocol without oral intraoperative antiplatelet therapy for endovascular treatment of ruptured intracranial aneurysms. *Journal of NeuroInterventional Surgery*.

[13] Zi-Liang W., Xiao-Dong L., Tian-Xiao L. (2017). Intravenous administration of tirofiban versus loading dose of oral clopidogrel for preventing thromboembolism in stent-assisted coiling of intracranial aneurysms. *International Journal of Stroke*.

[14] Roy D., Milot G., Raymond J. (2001). Endovascular treatment of unruptured aneurysms. *Stroke*.

[15] Mizutani T., Aruga T., Kirino T., Miki Y., Saito I., Tsuchida T. (1995). Recurrent subarachnoid hemorrhage from untreated ruptured vertebrobasilar dissecting aneurysms. *Neurosurgery*.

[16] Sughrue M. E., Saloner D., Rayz V. L., Lawton M. T. (2011). Giant intracranial aneurysms: evolution of management in a contemporary surgical series. *Neurosurgery*.

[17] Luzzi S., Gallieni M., Del Maestro M., Trovarelli D., Ricci A., Galzio R. (2018). Giant and very large intracranial aneurysms: surgical strategies and special issues. *Acta Neurochirurgica Supplement*.

[18] Algra A. M., Lindgren A., Vergouwen M. D. I. (2019). Procedural clinical complications, case-fatality risks, and risk factors in endovascular and neurosurgical treatment of unruptured intracranial aneurysms: a systematic review and meta-analysis. *JAMA Neurology*.

[19] Hassan T., Sultan A. E., Elwany M. N. (2011). Evaluation of balloon occlusion test for giant brain aneurysms under local anaesthesia. *The Neuroradiology Journal*.

[20] Ma Y., Zhang Y., Jiang J. (2019). Application and reliability of the superselective balloon occlusion test in the treatment of complex cerebral artery aneurysms: a report of 12 cases. *Journal of Clinical Neuroscience*.

[21] Sonmez O., Brinjikji W., Murad M. H., Lanzino G. (2015). Deconstructive and reconstructive techniques in treatment of vertebrobasilar dissecting aneurysms: a systematic review and meta-analysis. *American Journal of Neuroradiology*.

[22] Wang J., Jia L., Duan Z. (2019). Endovascular treatment of large or giant non-saccular vertebrobasilar aneurysms: pipeline embolization devices versus conventional stents. *Frontiers in Neuroscience*.

[23] Wang J., Liu X. F., Li B. M. (2017). Application of parallel stent placement in the treatment of unruptured vertebrobasilar fusiform aneurysms. *Journal of Neurosurgery*.

The article "Conservative Therapy vs. Endovascular Approach for Intracranial Vertebrobasilar Artery Trunk Large Aneurysms: A Prospective Multicenter Cohort Study" was retracted in 2023. Reasons: signs of a paper mill; suspected computer-generated content; unreliable results or conclusions; lack of ethics approval or compliance.

[24] Li M., Liang H., Wang J. (2020). Unfavorable outcomes related to endovascular treatment of giant vertebrobasilar aneurysms. *Frontiers in Neurology*.

[25] Mu S., Li C., Yang X. (2016). Reconstructive endovascular treatment of spontaneous symptomatic large or giant vertebrobasilar dissecting aneurysms: clinical and angiographic outcomes. *Clinical Neuroradiology*.

[26] Bhogal P., Perez M. A., Ganslandt O., Bäzner H., Henkes H., Fischer S. (2017). Treatment of posterior circulation non-saccular aneurysms with flow diverters: a single-center experience and review of 56 patients. *Journal of NeuroInterventional Surgery*.

[27] Kumar A., Dmytriw A. A., Salem M. M. (2020). Reconstructive vs deconstructive endovascular approach to intradural vertebral artery aneurysms: a multicenter cohort study. *Neurosurgery*.

[28] Zhang Y., Liang F., Zhang Y. (2019). Exploring the feasibility of pipeline embolization device compared with stent-assisted coiling to treat non-saccular, unruptured, intradural vertebral artery aneurysms. *Frontiers in Neurology*.

[29] Liang F., Zhang Y., Yan P. (2019). Predictors of periprocedural complications and angiographic outcomes of endovascular therapy for large and giant intracranial posterior circulation aneurysms. *World Neurosurgery*.

[30] Darsaut T. E., Darsaut N. M., Chang S. D. (2011). Predictors of clinical and angiographic outcome after surgical or endovascular therapy of very large and giant intracranial aneurysms. *Neurosurgery*.

[31] Nakatomi H., Kiyofuji S., Ono H. (2020). Giant fusiform and dolichoectatic aneurysms of the basilar trunk and vertebrobasilar junction-clinicopathological and surgical outcome. *Neurosurgery*.

[32] Flemming K. D., Wiebers D. O., Brown R. D. (2005). The natural history of radiographically defined vertebrobasilar nonsaccular intracranial aneurysms. *Cerebrovascular Diseases*.

[33] Cho D. Y., Kim B. S., Choi J. H., Park Y. K., Shin Y. S. (2019). The fate of unruptured intracranial vertebrobasilar dissecting aneurysm with brain stem compression according to different treatment modalities. *American Journal of Neuroradiology*.

